# The Efficacy of *Rosa damascena* on Liver Enzymes in Nonalcoholic Fatty Liver Disease: A Randomized Double-Blind Clinical Trial

**DOI:** 10.1155/2021/6628911

**Published:** 2021-08-12

**Authors:** S. Ali Al-Hadi Moravej, Asie Shojaii, Fataneh Hashem Dabaghian, S. Ferdows Jazayeri, S. Zahra Moravej, Ebrahim Khadem, Shahram Agah, Roshanak Ghods

**Affiliations:** ^1^Research Institute for Islamic and Complementary Medicine, Iran University of Medical Sciences, Tehran, Iran; ^2^Department of Persian Medicine, School of Persian Medicine, Iran University of Medical Sciences, Tehran, Iran; ^3^Department of Traditional Pharmacy, School of Persian Medicine, Tehran, University of Medical Sciences, Tehran, Iran; ^4^Ahvaz Jundishapur University of Medical Sciences, Department of Pharmacy, Ahvaz, Iran; ^5^Department of Traditional Medicine, School of Traditional Medicine, Tehran University of Medical Sciences, Tehran, Iran; ^6^Gastrointestinal and Liver Diseases Research Center, Iran University of Medical Sciences, Tehran, Iran

## Abstract

**Objective:**

This study aimed to appraise the potential effects of *Rosa damascena* preparation on nonalcoholic fatty liver disease (NAFLD).

**Design:**

In the randomized, double-blind placebo-controlled clinical trials, seventy-four patients with NAFLD were prescribed either 1 g *Rosa damascena* powder or placebo three times in a day for 12 weeks. All patients were provided the lifestyle modification instructions and recommended following them precisely. ALT, AST, FBS, and lipid profiles were measured at the baseline after 12 weeks of studying. The Mann–Whitney *U* test was correctly used to compare the changes of variables among the groups.

**Results:**

Seventy-two patients completed the study in two groups. Sixty-seven patients were men, and the mean ± standard deviation of age was 40.11 ± 9.05 years. The *Rosa damascena* group showed a considerable decrease in the serum ALT (23.83 ± 24.82 vs. 16.19 ± 27.41, *p*=0.042), waist circumference (99.73 ± 10.01 vs. 101.52 ± 8.84, *p*=0.003), triglyceride (TG) (186.29 ± 76.75 vs. 184.47 ± 73.05, *p*=0.001), cholesterol (167.47 ± 34.48 vs. 184.11 ± 33.54, *p*=0.001), low-density lipoprotein (LDL) (99.17 ± 28.66 vs. 107.52 ± 25.42, *p*=0.001), and elevation in serum high-density lipoprotein (HDL) (41.85 ± 6.56 vs. 39.20 ± 5.00, *p* < 0.007) compared to the control group. Improving fatty liver degree due to liver ultrasound was higher in the *Rosa damascena* group than the control group (*p*=0.001).

**Conclusion:**

*Rosa damascena* meaningfully improves liver function in NAFLD. Hence, it can be recommended along with lifestyle modification for these patients. Further studies are recommended with a larger sample size.

## 1. Introduction

Nonalcoholic fatty liver disease (NAFLD) remains the universal cause of chronic hepatic disorders [1]. Fatty droplets typically occupy the liver in the notable absence of other causes of hepatic steatosis [2]. However, its pathophysiology is not clearly known, but the multiple-hit hypothesis properly including steatosis, active inflammation, insulin resistance, active hormones promptly released from adipose tissue, specific nutrients, gut microbiota, genetic, and epigenetic factors were respectfully suggested [3]. There is a relationship between metabolic syndrome and NAFLD [4]. It is a silent disease, but without adequately treating it undoubtedly delivers two severe outcomes: (1) intrahepatic: steatohepatitis, cirrhosis, and hepatocellular carcinoma. (2) Extrahepatic: diabetes mellitus type 2, hyperlipidemia, hypertension, ischemic heart disease, and extrahepatic cancers, especially colorectal carcinoma [5]. Its most favorable treatment is lifestyle modification and drug prescription [6]. Antioxidant and immunomodulating drugs can treat this disease [7].

Persian medicine (PM) represents an ancient medical school which recommended some lifestyle modification methods (*Seteye-Zaroorieh*), herbal drugs, and hand practice or *a'amal-e-yadavee* such as massage and blood sampling methods (phlebotomy or fasd, cupping or hijamat, and leech therapy) for the treatment of disease [8]. Herbal preparation in PM was recommended for liver disease [9]. *Rosa damascena* is one of these cultivated plants that is planted and traditionally used in many countries such as Iran. The hepatoprotective effect of *Rosa damascena* is in terms of its components such as phenolic acid and flavonoid components [10]. Its petals have antioxidant and anti-inflammatory properties, and in animal studies, its effectiveness to clean the liver from accumulated triglycerides and prevent the inflammation of liver was shown [11]. Regarding PM principles, *Rosa damascena* has a pleasant odor; each aromatic herb reinforcing main organs such as the liver [12]. Since there is no clinical trial for the efficiency of *Rosa damascena* on NAFLD, this study was designated to show the *Rosa damascena* beneficial effect on liver enzymes and ultrasound grade in the patients with NAFLD.

## 2. Methods and Materials

### 2.1. Trial Design

This randomized, double-blind, placebo-controlled clinical trial was accomplished on two parallel groups of patients with NAFLD. Patients were appropriately allocated into two groups: intervention and placebo, by the block randomization method. The study protocol was approved by Medical Ethics Committee of Iran University of Medical Sciences (IR. IUMS REC.1398.406) and registered in Iran Clinical Trials Registry (ID: https://clinicaltrials.gov/ct2/show/IRCT20191006044994N1}).

### 2.2. Participants

The patients who met the inclusion criteria were enrolled in Behest Clinic affiliated with Iran University of Medical Sciences in Tehran, Iran. The study began on 1st March 2020 and ended on November 2020.

#### 2.2.1. Inclusion Criteria

  The patients (18–80 y) with nonalcoholic fatty liver disease
  Liver enzymes rising (AST > 38, ALT > 40)
  Ultrasound report grade 1 or 2 or three of fatty liver

#### 2.2.2. Exclusion Criteria

Acute or chronic liver disease, malignancy, pregnancy, uncontrolled diabetes mellitus, alcohol consumption, thyroid disease, psychological disorders, lactation, consumption of hepatotoxic drugs within the past 6 months, consumption of drugs which can affect the assessed biochemical tests of study within the previous 3 months (e.g., metformin, vitamin E, oral contraceptive pills, statins, and glucocorticoids), heart and adrenal insufficiency, and that did not want to willingly participate.

### 2.3. Intervention

After signing a written informed consent and taking a complete history of patients at the start of the study, they were randomly divided into two groups as case and control. Patients in both groups were given dietary recommendations due to classical medicine and recommended walking at an average speed for 40 minutes daily. The patients in the intervention group and who were in the placebo group received two capsules, each containing 500 mg of petal powder of *Rosa damascena* or toast powder, three times in a day, 30 minutes before a meal or 2 hours after the meal. Both groups were carefully followed for 12 weeks. *Rosa damascena* and placebo capsules were packaged in similar containers and labeled accordingly. Consumption of less than 80% of the drug during the trial was considered as drug intolerance, and the patient was excluded from the trial.

For concealment, sealed envelopes were used, so that the distinct number was recorded on similar envelopes. The drug and placebo were coded in similar capsules and identical packages with the same color and aroma. The patient and researcher were unaware of how the drug or placebo was coded.

This study aimed to appraise the potential effects of *Rosa damascena* preparation on liver enzymes in nonalcoholic fatty liver disease (NAFLD), especially ALT enzyme, at the beginning and the end of the 12th week of study.

Upon entering the study and completing it, all participants were evaluated in terms of blood pressure, waist circumference, height, and weight. A standard mercury calibrated sphygmomanometer was used to measure the blood pressure. Participants rested for 15 minutes, and in a sitting position, blood pressure was taken from their right hand. A rubber meter was properly used to accurately measure the waist circumference in the upright position. A standard meter and an accurate scale were properly used to accurately measure the height and weight. BMI was calculated due to standard formula: BMI = weight (kg)/height (m^2^).

All these measurements were performed by a trained nurse. Blood samples were collected from the right hand of all participants after 12 hours of fasting. Complete blood count (CBC), biochemical (FBS, BUN, Cr, total cholesterol, TG, HDL, LDL, AST, and ALT) tests, and U/A (S. G) were precisely measured at weeks 0 and 12. For a significant amount of liver enzymes, photometric assay, and accurate measurement of blood glucose and other biochemical tests, an enzymatic colorimetric method using the standard kits (Pars Azmoun Company, Iran) was properly used. An experienced radiologist satisfactorily performed a liver ultrasound at the marked beginning and the end of controlled study.

#### 2.3.1. Fatty Liver Score according to Ultrasound Grades

1. Mild increased hepatic echogenicity with normal visualization of diaphragm and intrahepatic vessels
2. Moderate increased hepatic echogenicity with mildly impaired visualization of diaphragm and intrahepatic vessels
3. Severe increased hepatic echogenicity and poor or nonvisualization of diaphragm and intrahepatic vessels.

### 2.4. Drug and Placebo Preparation

*Rosa damascena* was collected from Marand city located in East Azerbaijan province and authenticated by a botanist from School of Pharmacy, Tehran University of Medical Science, Tehran, Iran (voucher no: pmp 584). The rose petals were carefully separated from the sepals and, after drying and crushing, were placed in 500 mg gelatin capsules. *Rosa damascena* capsules were used for better acceptance in patients. Placebo powder (toasted flour) was also filled in 500 mg capsules similar to *Rosa damascena* capsules.

### 2.5. Sample Size

Sufficient sample size was carefully calculated by proper utilization of pilot study information and the standard formula for accurately comparing two means and correctly observing 20 units of essential ALT difference between two specific groups with an alpha error of 0.05, power 80%, and with the expectation of 20% potential loss to proper follow-up. Ultimately, 74 patients (37 persons in each group) were enrolled.

### 2.6. Statistical Analysis

The patients with medication compliance as 80% or more entered the analysis. Data were carefully analyzed by SPSS software (version 17). The specific Kolmogorov–Smirnov test promptly confirmed the standard distribution of variables. The effective mean ± standard deviation or number and frequency percentage were properly used to typically describe the variables. The chi-square or Fisher exact test and independent *t*-test or Mann–Whitney *U* test were typically used to accurately compare the independent variables between two groups. Within-group analyses were typically performed using the Wilcoxon signed ranks test. *P* values less than 0.05 were considered statistically significant.

### 2.7. Safety Measures and Adverse Events

At the beginning of the study, a form was provided to patients in each group to record possible drug side effects such as gastrointestinal symptoms, constipation, diarrhea, and the effect on libido. CBC, BUN, and serum creatinine levels at weeks 0 and 12 were normal, and there were no significant changes in both groups. There was no report of severe adverse events in any patients.

## 3. Results

234 patients were enrolled, and 160 subjects who had not met the inclusion criteria were excluded. Seventy-four patients who met the inclusion criteria and agreed to participate in the study were divided into two groups. Thirty-seven patients were assigned to the intervention group and 37 patients to the control group. From each group, one individual was excluded in terms of COVID-19. In total, seventy-two cases completed the study. Thirty-six patients were in the *Rosa damascena* group and 36 patients in the placebo group (Figure 1).

The baseline characteristics of studying groups are summarized in Table 1. At the baseline, the frequency of all the primary and secondary outcome variables was statistically identical among groups except systolic blood pressure. To control the confounding effect of baseline systolic blood pressure, percent changes of systolic blood pressure were compared among groups. Regarding demographic characteristics, the mean age of participants was 41.5 ± 9.85 and 38.7 ± 8.07 years in the intervention and control groups, respectively. There were no significant differences in baseline demographic data and age, gender, and BMI between the two groups (Table 1).

Regarding laboratory indices, there were no significant differences in FBS, grade of NAFLD in ultrasound, ALT and AST, lipid profiles, and urine-specific gravity levels between two groups at the beginning of study (Tables 1 and 2).

Significant differences were observed due to baseline systolic blood pressure (*p* value = 0.004) (Table 1).

Following the patient in both groups, compliance with lifestyle did not indicate any significant differences among the groups. We followed the patients in both groups in terms of compliance with lifestyle modification every week and recalled them to do the diet and exercise instructions. Weight loss among 3–5% during 12 weeks was considered to assess the compliance of life and exercise modification between two groups; at the end of study, the weight change in the participants of two blocs was about 3–5% (Table 1).

### 3.1. Primary Outcome

Analyzing the results after 12 weeks reflected that there was a substantial reduction in the serum ALT levels in both groups. The percent decrease of ALT was significantly higher in the *Rosa damascena* group than in the control group (*p*=0.042) (Table 1).

### 3.2. Secondary Outcomes

Except HDL, lipid profiles significantly decreased in the intervention group (TG, Chol, and LDL, *p* > 0.001), but HDL significantly increased in the intervention group (*p* < 0.007) (Table 1).

In both groups, the anthropometric factors such as weight, BMI, and WC reduced after 12 weeks, but WC was significantly decreased in the intervention group (*p* < 0.003) (Table 1).

Diastolic pressure significantly decreased in the intervention group (*p*=0.001). Platelet count and SG were significantly decreased in the intervention group (platelet, *p* > 0.002 and SG, *p* > 0.001) (Table 1).

Moreover, there was a significant reduction in NAFLD grade in ultrasound in the *Rosa damascena* group compared to the placebo over the studying period (*p* value = 0.001) (Table 2).

## 4. Discussion

This study is the first randomized clinical trial investigating the effect of *Rosa damascena* petals on NAFLD. In this double-blind clinical trial, ordinary consumption of 3 g (two capsules, three times in a day) of *Rosa damascena* petal capsules for 12 weeks were compared to the placebo. There was no considerable gap in BMI among two groups. Various investigations indicated that 5–10% weight loss is considered for dietary consumption and exercise efficiency to improve the NAFLD [13]. Weight loss percent was less than 5% in both groups (Table 1).

The results showed that *Rosa damascena* could reduce liver enzymes (especially ALT), lipid profile, and blood pressure, meaningfully improve metabolic syndrome components, and increase urine SG.

Considering multihit hypothesis, steatosis persists as the first event in the pathogenesis of NAFLD. Davoodi et al. showed that *Rosa damascena* could significantly reduce the final liver fat accumulation, TG, TC, and LDL-C serum concentrations, and hepatic enzymes in an experimental study [11]. Active inflammation is the second notable event in NAFLD pathogenesis [3]. *Rosa damascena* organic compositions such as flavonoids and phenols naturally have anti-inflammatory outcomes and severely inhibit destructive effects of active inflammation on the liver. Flavonoids components inhibit de novo lipogenesis and modulate intestinal microbiota imbalance [10].

Previous studies indicated that NAFLD increases hypertension, following cardiovascular diseases. Proper treatment of NAFLD can reduce cardiovascular disease incidence [14]. *Rosa damascena* naturally has cyanidin‐3‐O‐B glucosides which efficiently remain as an antihypertensive agent in terms of inhibiting angiotensin‐converting enzyme [15]. Many patients reported less depression and better sleep at the end of the study. These effects may be due to strengthening the vital organs, such as the brain, heart, and liver [16].

This study showed that urine-specific gravity increases after *Rosa damascena* consumption. Specific gravity represents an expression of urine concentration in terms of density. Fluid density critically depends on the sufficient number of solute particles present and their relative mass. Specific gravity measurement is used to reasonably assess the measurable quantity of solutes present in urine. It accurately reflects the ability of functioning kidneys to naturally produce the effective urine [17].

Another outcome was a reduction in the platelet count. Flavonoids contain many components, such 4-methylcatechol that is normally formed by human microflora. It poses a strong antiplatelet effect which can typically decrease the elevated incidence of cardiovascular diseases. This information can help explain the antiplatelet potential of orally given flavonoids containing formulas such as *Rosa damascena* [18].

In brief, after a favorable review of properties as mentioned above of *Rosa damascena*, it is typically recommended that before doing liver-destroying drugs such as halothane, advised patient should employ *Rosa damascena* for a certain period and typical dose along with lifestyle modification. This effect is due to synchronous properties of antioxidant activity and liver protector of *Rosa damascena*.

The safe dose of powder of *Rosa damascena* is up to 12 g [12]. Winther et al. found that the effective dose of *Rosa damascena* when used as the dried powder is 5 g per day [19]. We use 3 g or two 500 mg capsules three times a day. No significant reduction in the additional variables such as FBS might were due to the low doses of preparing in this study, and higher dosage or other types of preparation or more prolonged treatment time might be needed.

There were some limitations such as the short duration of the study and using *Rosa damascena* as a capsule for better acceptance in the patients (in the PM, its decoction form is recommended). The effect of *Rosa damascena* on liver histology (liver biopsy) was unstudied because it was quite invasive. The prevalence of the COVID-19 pandemic prevents the patients from participating in the study or causes them to leave the study.

## 5. Conclusion

This study showed that *Rosa damascena* petals powder consumption with a daily dose of 3 g for 12 weeks improved ALT enzyme, reduced fatty liver grade in ultrasound (Table 2), and better metabolic syndrome components in informed patients with NAFLD. Regarding the cost-effectiveness and availability of *Rosa damascena* and the lack of any reports for serious complications of this plant using, *Rosa damascena* can be recommended in patients with NAFLD. Further research with larger sample size and long‐term follow‐ups of patients, further research with a larger sample size can provide a stronger document about the usage of *Rosa damascena* as complementary medicine to treat the NAFLD.

## Figures and Tables

**Figure 1:** Participant flow.

**Table 1:** Amount variables at different times.

Variables	Group	Baseline mean ± SD	*P* value	After 12 weeks mean ± SD	*P* value	Percent change mean ± SD	*P* value
BMI (kg/m^2^)	Rd	29.68 ± 3.66	0.064	28.46 ± 3.62	0.640	4.08 ± 3.96	0.102
	Placebo	30.05 ± 3.88		29.22 ± 3.85		2.71 ± 3.18	
WC (cm)	Rd	103.69 ± 10.64	0.967	99.73 ± 10.01	0.424	3.75 ± 2.76	0.003
	Placebo	103.79 ± 8.89		101.52 ± 8.84		2.14 ± 2.71	
ALT (IU/L)	Rd	69.05 ± 25.38	0.364	45.22 ± 19.45	0.262	31.52 ± 27.3	0.042
	Placebo	66.41 ± 25.24		50.22 ± 20.60		18.66 ± 29.62	
AST (IU/L)	Rd	1.82 ± 38.38	0.937	30.19 ± 9.83	0.787	13.40 ± 33.86	0.166
	Placebo	37.44 ± 16.03		31.83 ± 12.60		11.33 ± 20.59	
Systolic BP (mmHg)	Rd	125.47 ± 13.47	0.004	118.52 ± 11.33	0.18	5.33 ± 4.18	0.001
	Placebo	113.08 ± 11.70		113.47 ± 11.62		−0.395 ± 3.00	
Diastolic BP (mmHg)	Rd	82.47 ± 12.17	0.97	82.47 ± 11.21	0.717	3.90 ± 7.78	0.001
	Placebo	82.60 ± 7.20		82.60 ± 7.51		0.22 ± 3.85	
FBS (mg/dl)	Rd	108.85 ± 26.31	0.251	103.11 ± 26.77	0.713	3.12 ± 16.14	0.103
	Placebo	100.08 ± 25.12		103.94 ± 40.7		−3.42 ± 15.89	
TG (mg/dl)	Rd	225.44 ± 121.16	0.112	186.29 ± 76.75	0.764	9.61 ± 35.11	>0.001
	Placebo	190.70 ± 100.29		184.47 ± 73.05		−3.67 ± 25.55	
Cholesterol (mg/dl)	Rd	199.23 ± 30.81	0.214	167.47 ± 34.48	0.048	14.66 ± 18.95	>0.001
	Placebo	189.14 ± 35.29		184.11 ± 33.54		2.13 ± 8.01	
HDL (mg/dl)	Rd	36.82 ± 7.22	0.961	41.85 ± 6.56	0.044	−14.94 ± 13.03	0.007
	Placebo	35.85 ± 4.06		39.20 ± 5.00		−9.8312.65	
LDL (mg/dl)	Rd	112.91 ± 28.12	0.112	99.17 ± 28.66	0.208	19.97 ± 20.83	>0.001
	Placebo	112.08 ± 27.26		107.52 ± 12.60		3.28 ± 9.44	
Platelet (mm^3^ × 10^3^)	Rd	257.86 ± 43.69	0.333	237.36 ± 43.99	0.768	7.53 ± 9.11	>0.002
	Placebo	240.40 ± 78.53		238.25 ± 54.21		0.05 ± 17.88	
Urine SG	Rd	**1019.61** **±** **7.04**	0.276	1025.79 ± 5.82	0.027	−0.60 ± .54	>0.001
	Placebo	1021.47 ± 8.86		1022.02 ± .75		−0.05 ± 5.17	

BMI, body mass index; WC, waist circumference; ALT, alanine aminotransferase AST, aspartate aminotransferase; FBS, fasting blood sugar; TG, triglyceride, HDL, high-density lipoprotein, LDL, low-density lipoprotein, SG, specific gravity, minus means to increase; Mann–Whitney *U* test.

**Table 2:** The ultrasound changes at different times.

Ultrasound grade	Baseline		*P* value	After 12 weeks		*P* value
	Rd = 36	Placebo = 36		Rd = 35	Placebo = 36	
Grade 1	7	8	0.635^*∗∗*^	25	9	0.001^*∗∗*^
Grade 2	27	24		10	22	
Grade 3	2	4		0	5	

^*∗∗*^Person chi-square test.

## Data Availability

The data used to support the findings of this study are included within the article.
